# Serum Metabolomics of Benign Essential Blepharospasm Using Liquid Chromatography and Orbitrap Mass Spectrometry

This article has been retracted.

**DOI:** 10.1155/2022/6876327

**Published:** 2022-11-18

**Authors:** Han Zhao, Wushuang Wang, Tong Lin, Lan Gong

**Affiliations:** ^1^Department of Ophthalmology, Eye, Ear, Nose, and Throat Hospital of Fudan University, Shanghai 200000, China; ^2^Laboratory of Myopia, NHC Key Laboratory of Myopia (Fudan University), Chinese Academy of Medical Sciences, Fudan University, Shanghai 200000, China; ^3^Shanghai Key Laboratory of Visual Impairment and Restoration, Fudan University, Shanghai 200000, China

## Abstract

**Background:**

Benign essential blepharospasm (BEB) is a form of focal dystonia that causes excessive involuntary spasms of the eyelids. Currently, the pathogenesis of BEB remains unclear. This study is aimed at investigating the serum metabolites profiles in patients with BEB and healthy control and to identify the mechanism and biomarkers of this disease.

**Methods:**

30 patients with BEB and 33 healthy controls were recruited for this study. We conducted the quantitative and nontargeted metabolomics analysis of the serum samples from 63 subjects by using liquid chromatography and Orbitrap mass spectrometry (LC-Orbitrap MS). Multivariate statistical analysis was performed to detect and identify different metabolites between the two groups. The Kyoto Encyclopedia of Genes and Genomes (KEGG) and receiver operating characteristic (ROC) curve analysis of the altered metabolites were performed.

**Results:**

A total of 134 metabolites were found and identified. The metabolites belonged to several metabolic pathways including phenylalanine metabolism, phenylalanine, tyrosine and tryptophan biosynthesis, arginine biosynthesis, linoleic acid metabolism, tryptophan metabolism, aminoacyl-tRNA biosynthesis, sphingolipid metabolism, glycosphingolipid biosynthesis, leucine and isoleucine biosynthesis, and vitamin B6 metabolism. Eight metabolites were identified as the potential biomarkers.

**Conclusions:**

These results demonstrated that serum metabolic profiling of BEB patients was significantly different from healthy controls based on LC-Orbitrap MS. Besides, metabolomics might provide useful information for a better understanding of BEB.

## 1. Introduction

Benign essential blepharospasm (BEB) is an adult-onset focal dystonia marked by excessive involuntary spasms of the orbicularis oculi muscle as well as other motor symptoms such as elevated blink frequency and apraxia of eyelid opening. As the disease progresses, dystonia in about two-thirds of these patients will expand to adjacent muscle sites, including the oromandibular and cervical muscles, within five years of BEB initiation [1]. The mean annual incidence of BEB was reported as 0.10 in a recent population-based retrospective analysis [2]. BEB is more frequent in women, and the peak incidence of them frequently appeared in their fifth and sixth decades [3]. The epidemiological study showed that the majority of BEB cases were considered sporadic, with just 20–30% of cases having a familial history [4]. As the symptoms progress, it may become difficult to open the eyes or even induce functional blindness, resulting in functional impairment at work and in everyday life as well as a reduction in quality of life [5].

Research on BEB has gotten a lot of attention, and there has been a lot of development. While the specific mechanism of BEB remains vague, however anomalies in both the basal ganglia and cortical function have been blamed. Furthermore, both genetic and metabolic variables are implicated in BEB progression [1, 6]. The metabolic alterations were a potential factor involved in the pathogenesis of BEB. Suzuki et al. found that the glucose metabolism level was higher in both sides of the posterior striate cortex and extrastriate cortex of patients with BEB when compared with normal subjects by using positron emission tomography. During the study, the severity of BEB was also linked to thalamic glucose metabolism [7]. Mostofsky et al. also reported that essential fatty acids administration could alleviate the eye blinking rate in the dopamine depletion-induced blepharospasm rat model [8]. In addition, there was a significant decrease in serum calcium levels in the BEB group compared with the healthy group [9].

Metabolomics is a relatively emerging discipline that analyzes the intermediary and final products of the metabolic pathways within an organism; therefore, it is possible to reflect the alterations in these compounds under any pathological stimulation, genetic effect, or physiological condition. Nontargeted metabolomics analysis, which has been widely utilized in clinical research, may identify metabolites in a variety of materials, including tear fluid, urine, and serum [10]. In addition, metabolomics has a particular advantage over other technologies including genomics, transcriptomics, and proteomics in that it could provide a global phenotype of metabolic changes. This approach is now being utilized to find evidence of major changes in metabolites such as amino acids, lipids, and neurotransmitters in dystonia-related diseases [11–13]. There have been no reports of using metabolomics to uncover pathogenic aspects or diagnostic biomarkers in BEB patients, suggesting that this novel technology must be employed to identify probable biomarkers of BEB as well as explore the disease's pathogenesis and treatment approaches.

In the present study, we have performed a study to determine the metabolic characteristics and networks in the serum of patients with BEB based on liquid chromatography and Orbitrap mass spectrometry (LC-Orbitrap MS). The purpose was to investigate the serological biomarkers for BEB diagnosis and the pathogenesis of the BEB.

## 2. Materials and Methods

### 2.1. Standard Protocol Approvals and Patient Consents

The protocols of this study were approved by the Ethics Committee of Eye, Ear, Nose, and Throat Hospital of Fudan University. The informed consent process was adhering to the tenets of the Helsinki Declaration, and all BEB subjects and healthy individuals signed the informed consent forms.

### 2.2. Study Participants Collection

In total, 30 BEB patients were enrolled from the Department of Ophthalmology of Eye, Ear, Nose, and Throat Hospital of Fudan University from July 2021 to December 2021. To prevent any diagnostic bias, all individuals underwent a routine ophthalmology examination by two ophthalmologists. Inclusion criteria included patients who were 20 years of age or older with the diagnosis of BEB by experienced ophthalmologists or neurologists. The following exclusion criteria were applied to all BEB subjects: (1) any ocular abnormalities such as conjunctivitis, keratitis, glaucoma, or uveitis; (2) any systemic diseases such as hypertension, hyperlipidemia, heart disease, diabetes, metabolic diseases, or hematological diseases; (3) topical or systemic medications. The severity and frequency of blepharospasm were evaluated by using the Jankovic rating scale (JRS) [14]. The functional impairments in daily life activities of BEB in all patients were accessed according to the blepharospasm disability index (BSDI). Disease duration was determined in months from the beginning of symptoms to the date of the examination. In the control group, another 33 healthy individuals without BEB were included, and their serum was taken with normal clinical blood draws.

### 2.3. Samples Preparation

The 2 mL vacuum blood collection tube was used to collect a whole blood sample from each participant during another normal blood testing. Tubes were then centrifuged for 5 minutes (3000 rpm/min, 4°C) to remove the blood cells, and the supernatant was transformed into 2 mL cryogenic vials (NEST Biotechnology) and promptly stored at -80°C before metabolomic analysis.

For LC-Orbitrap MS analysis, each 100 *μ*L of serum was thawed at 4°C and mixed with a 300 *μ*L solution of cold methanol/phenylalanine. After vortexing for 2 minutes, the samples were then centrifuged for 10 minutes (13000 rpm/min, 4°C) and obtained 200 *μ*L supernatants.

### 2.4. LC-Orbitrap MS Analysis

The UHPLC system was coupled to an Orbitrap MS (Waters Corp., Milford, MA, USA) equipped with an electrospray ionization source, operating in positive or negative ionization mode, with a mass resolution of 70,000 and m/z of 200. The full scan mass resolution was 17500 at m/z 200 using data correlation (dd-MS2, TopN = 10) MS/MS mode. Scanning range: 100-1500. The chromatographic conditions were as follows: the injection volume was 2 *μ*L, the column temperature was 25°C, the flow rate was 0.35 mL/min, and the mobile phases were 0.1% formic acid aqueous solution (solution A) and 0.1% formic acid acetonitrile solution (solution B). The optimized chromatographic gradient is as follows: 0-2 min, 5% in solution B; 2-10 min, 5%-95% in solution B; 10-15 min, 95% in solution B; 15-18 min, 5% in solution B. The following parameters were used for mass detection in both positive and negative ion modes: scan range, m/z 80-1000; drying gas (N_2_) flow rate, 11 L/min; gas temperature, 350°C; pressure of the nebulizer gas, 45 psig; Vcap, 4000 V (-3000 V). Data were acquired in centroid mode using Thermo Excalibur 2.2 software (Thermo Fisher Scientific, MA, USA).

### 2.5. Statistical Analysis

Data were acquired using Thermo Xcalibur 2.2 software (Thermo Scientific, San Jose, USA). Peak calibration and extraction were performed using composite discovery software (Thermo Fisher Scientific). Data tables were imported into SIMCA-P 13.0 (Umetrics AB, Umea, Sweden) for multivariate statistical analysis. An unsupervised principal component analysis (PCA) was used to assess the overall trend of separation between these samples. Differential metabolites were screened by partial least squares-discriminant analysis (PLS-DA). According to the PLS-DA model, variables with variable importance in the projection (VIP) value greater than 1.0 were selected, SPSS Statistics 18.0.0 was used to perform a two-tailed Student *t*-test, and *p* < 0.05 was considered statistically significant. Multiple-test adjustment was performed with Bonferroni correction. To identify these potential biomarkers, accurate ion masses were entered into the Human Metabolome Database (HMDB), Metlin, MoNA, and MassBank databases to match accurate molecular weights and automatically search for MS1/MS2 fragment ions. Finally, to determine the structure of the compound, we used our library of internal standard metabolites, matching accurate masses, fragment ion masses, and retention times. Pathway enrichment analysis was performed using the Kyoto Encyclopedia of Genes and Genomes (KEGG) database and metabolic analysis (https://www.metaboanalyst.ca/). The diagnostic power of the biomarkers was assessed using the area under the (ROC) curve.

## 3. Results and Discussion

### 3.1. Baseline Characteristics of the Study Subjects

The workflow of our study is shown in Figure 1. The baseline characteristics of the study subjects are shown in Table 1. Totally 63 participants, including 30 BEB subjects and 33 control subjects were recruited. Differences in age, gender, and BMI were not significant between BEB patients and controls (*p* > 0.05).

### 3.2. Total Ion Chromatogram and Untargeted Metabolomics Analysis of Serum Samples

Figures 2(a) and 2(b) show a representative total ion chromatogram (TIC) data from the serum of the BEB group and control group. The good overlap of retention time of each main chromatographic peak in both positive and negative ionization modes proved the LC-Orbitrap MS system's exceptional stability and repeatability throughout the procedure. To evaluate the serum level of altered metabolites in BEB, we performed a nontargeted metabolomics analysis of 63 serum samples by LC-Orbitrap MS. Figures 2(c) and 2(d) show PCA score plot for the BEB, control, and quality control (QC) groups. In both positive and negative ionization modes, a high degree of aggregation of the QC groups was identified, indicating the high stability and good repeatability during the whole sequence of the BEB and control groups. The PLS-DA was carried out to determine the metabolites pattern changes in the BEB and control groups. The PLS-DA plot scores (Supplementary Figures 1A and 1B) revealed a strong distinction between the BEB and control groups. The permutation analysis of the PLS-DA plot also indicated a high validity and stability in both the BEB group and control group (Supplementary Figures 1C and 1D).

### 3.3. Differentiating Metabolite Identification

According to the criteria of VIP > 1 and *p* < 0.05, volcano plot analysis was been applied to determine significant differences of the metabolites between the two groups. The red or green dots depict metabolites that substantially changed between BEB and control groups under positive ionization mode (Figure 3(a)), negative ionization mode (Figure 3(b)), and combination mode (Figure 3(c)). The serum of the BEB group was then compared to that of the control group, yielding 134 differently expressed metabolites, as shown in Supplementary Table 1. To further determine the altered metabolites between the BEB group and the control group, a clustering heatmap showed altered metabolites under the positive ionization mode between these two groups (Figure 4(a)). We also explored the metabolic differences between BEB patients and controls under negative ionization mode of electrospray ionization.  Figure 4(b) shows that 41 metabolites were identified between two differentiated clusters. On the other hand, Figure 4(c) shows metabolic differences between BEB patients and controls under combination mode. Pair-wise Spearman analysis was used to analyze the correlation coefficient between serum differential metabolites and clinical parameters (Figure 4(d)). Significant correlations were also observed between the course of disease and penta-L-phenylalanine. However, no significant correlation was observed between serum differential metabolites and JRS or BSDI.

To identify the serum level of nontargeted metabolomics profiles in course of BEB, we performed a nontargeted metabolomics analysis of BEB patients and their control at 0-12 months, 13-24 months, and more than 24 months. At 0-12 months, 57 metabolites were significantly altered, including 36 upregulated metabolites and 21 downregulated metabolites (*p* < 0.05). At 13-24 months, there were 29 metabolites significantly changed (*p* < 0.05). Among them, 22 were increased and 7 were decreased. Moreover, 46 metabolites were significantly changed in the BEB group at more than 24 months. 32 metabolites were significantly increased, whereas 14 metabolites were significantly decreased (Supplementary Table 2).

### 3.4. KEGG Analysis of Differential Plasma Metabolites

KEGG pathway enrichment studies were done based on the changed metabolites in both positive and negative ionization modes of electrospray ionization to investigate the pathways implicated in these altered serum metabolites. Phenylalanine metabolism, phenylalanine, tyrosine and tryptophan biosynthesis, arginine biosynthesis, linoleic acid metabolism, tryptophan metabolism, aminoacyl-tRNA biosynthesis, sphingolipid metabolism, glycosphingolipid biosynthesis, leucine and isoleucine biosynthesis, and vitamin B6 metabolism were the top 10 enriched pathways, as illustrated in Figure 5.

### 3.5. Biomarker Identification of Important Metabolites

To further screen the potential metabolic indicators in serum samples of BEB patients, ROC curve analysis was performed to identify the sensitivity and specificity of significantly altered metabolites. ROC curve analysis was considered the candidate diagnostic biomarker for BEB according to an area under the ROC curve (AUC) >0.8. PC (18 : 1(11Z)/24 : 1(15Z)), TG (16 : 0/19 : 0/20 : 0) [iso6], PC (O-22 : 0/22 : 3(10Z,13Z,16Z)), PC (16 : 0/24 : 1(15Z)), PS (16 : 0/22 : 1(11Z)), hexadecyl phosphorodichloridate, methionine sulfoxide, and icotidine all had AUC values of 1.000, 0.991, 0.981, 0.978, 0.915, 0.835, 0.824, and 0.801, respectively (Figure 6, Table 2).

## 4. Discussion

BEB is regarded as a common movement disorder worldwide characterized by increased activity of the orbicularis oculi muscle and other muscles around the eyelid. Although blepharospasm was first reported 80 years ago, the etiological mechanisms remain not clear. There is an urgent need to investigate the etiological mechanisms or find a potential diagnostic biomarker in BEB patients.

The primary aim of this study was to systematically analyze the serum metabolites of BEB. Therefore, we examined altered serum metabolites profiles in 30 subjects with BEB and 33 age-matched healthy controls based on LC-Orbitrap MS. A significant distinction between the BEB patients and healthy individuals was accomplished using multivariate statistical analysis. The potential metabolic indicators responsible for the separation of BEB and the control groups were revealed by the loading plots from the PCA in positive and negative ionization modes. 134 metabolites exhibited significant differences between the two groups, according to the *p* values of the independent test. Moreover, these altered metabolites with linked to the metabolic pathways of phenylalanine metabolism, phenylalanine, tyrosine and tryptophan biosynthesis, arginine biosynthesis, linoleic acid metabolism, tryptophan metabolism, aminoacyl-tRNA biosynthesis, sphingolipid metabolism, glycosphingolipid biosynthesis, leucine and isoleucine biosynthesis, and vitamin B6 metabolism were identified as preliminary. In addition, we compared metabolite expression levels between patients with different disease courses. Some lipid subclass and amino acids and their derivatives were found to be significantly changed at 13-24 months and more than 24 months, respectively. These results suggest that BEB development is accompanied by a metabolomic change of amino acids from the lipid subclass and their derivatives. It is also interesting to observe that the metabolomic change in patients with BBE more than 24 months indicated that BEB may have a long-term effect on the metabolite profile. These metabolites can serve as potential biomarkers or monitoring indicators for different disease processes.

Extensive studies have indicated that movement disorders such as focal dystonia and Parkinson's disease linked to oxidative stress [15]. However, the mechanisms responsible for oxidative stress in BEB are not fully understood. In our study, tryptophan, the antioxidants amino acid, and the production of tyrosine and dihydroxyindole, were markedly decreased in BEB group. Tryptophan can modulate the function of antioxidant enzymes, such as glutathione s-transferase, and tyrosine, an important antioxidant, may reduce oxidative damage by lowering ferryl hemoglobin levels [16]. In addition, previous study suggested the reduced tryptophan levels may be linked to chronic inflammation in white matter [17]. The higher L-kynurenine/tryptophan ratio found in this study suggests that the activation of oxidative stress or inflammation is considerably boosted in BEB (Supplementary Figure 2). These findings suggest that in BEB, downregulation of the tyrosine and tryptophan biosynthesis-related pathway may disturb the antioxidative system.

Phosphatidylcholine (PC) is an important metabolite in the nervous system. PC synthesis was increased in neuronal differentiation [18]. PC's involvement in membrane fluidity is especially critical for neuronal homeostasis by preventing the protein from aggregating [19]. The balance of lipid content as well as lipid-to-protein proportions can be disrupted and therefore a disease risk factor for Parkinson's disease [20]. PC also affects the characteristics of peripheral neurotoxicity. PC may promote the development of neurons and decrease oxidative stress by increasing antioxidant levels [21]. PC is mainly synthesized and abundant in the endoplasmic reticulum, and it synthesize might occur in endoplasmic reticulum stress [22]. However, as shown in the context of obesity and a mouse model of muscular dystrophy, an increase in PC can also activate endoplasmic reticulum stress responses, implying that PC plays a key role in endoplasmic reticulum stress [23, 24]. Moreover, endoplasmic reticulum stress may contribute to the deficits in neuroplasticity and motor function in dystonia [25]. In our study, serum level of PC (16 : 0/24 : 1(15Z)) and PC (18 : 1(11Z)/24 : 1(15Z)) were significantly increased in the BEB group, while PC (14 : 0/18 : 2(9Z,12Z)), PC (14 : 0/22 : 6(4Z,7Z,10Z,13Z,16Z,19Z)), PC (O-18 : 1(9Z)/16 : 0), and PC (14 : 1(9Z)/24 : 1(15Z)) were decreased in BEB patients, which indicates dysfunction of PC subclasses. In this study, LysoPC (16 : 0/0 : 0) was decreased in BEB patients, while LysoPC (22 : 5(4Z,7Z,10Z,13Z,16Z)/0 : 0), LysoPC (0 : 0/16 : 0), and LysoPC (22 : 4(7Z,10Z,13Z,16Z)/0 : 0) were increased in BEB. Due to disruption of the cell membrane and the presence of inflammation with BEB, the dysfunction of LysoPCs caused changes in energy metabolism. This might be a possible mechanism of BEB and remains further studied.

Phosphatidylethanolamine (PE) is the main part of phospholipid in human plasma. Phospholipids are the important components of the cell membrane surfactants and affect various membrane functions, including cell membrane formation, activation of several membrane-bound enzymes, cell membrane recognition, and signal transduction [26]. Moreover, studies have confirmed that loss of PE asymmetry in the cell membrane can activate a multitude of pathophysiological processes, such as apoptosis and necrosis [27]. In addition, one of the most important consequences of PE abnormalities is the change in energy metabolism in the endoplasmic reticulum leading to endoplasmic reticulum stress in Parkinson's disease [28]. Wortmann et al. also found a PE remodeling-related gene and gene mutation could impair mitochondrial function and cause dystonia [29]. Our results indicated PE metabolism disorder in patients with BEB as compared to the control group, which was evidenced by altered levels of PE-NMe (14 : 1(9Z)/20 : 1(11Z)), LysoPE (0 : 0/22 : 5(4Z,7Z,10Z,13Z,16Z)), PE (18 : 0/20 : 4(5Z,8Z,11Z,14Z)), and PE (18 : 1(9Z)/0 : 0). However, PE is not only affected by daily diet but also by systemic metabolism, so it is difficult to standardize the diet of all participants at the time of enrollment, so the role of PE in BEB is still not known and remains further study.

Phosphatidylserine (PS) plays a key role in the function and structure of the human nervous system. PS accounts for 13%-15% of the total phospholipids in the adult cerebral cortex [30]. PS is a key compound required for activating several critical signaling pathways in the membrane of plasma, such as the Akt and Raf-1 signaling pathways, which are involved in neuronal survival, process development, and synaptogenesis [31]. PS also plays a role in modulating AMPA glutamate receptors [32]. In the synapses, PS mediates calcium-dependent membrane fusion among synaptic vesicles and the target membrane, which is regulated by synaptotagmin and the soluble N-ethylmaleimide-sensitive factor attachment protein receptor complex, which is necessary for exocytosis [33]. A recent study showed significantly decreased levels of serum calcium in the BEB group compared with the healthy group [9]. PS synthase in the neurons was also shown to be aberrant in Parkinson's disease [34]. Blepharospasm is common in Parkinson's disease [35]. In this study, PS (16 : 0/22 : 1(11Z)) was increased in the BEB group compared with the control group, while PS (O-16 : 0/13 : 0) and PS (O-18 : 0/0 : 0) were decreased in the BEB groups. The roles of serum PS subclasses in BEB patients have not been fully elucidated. The possible mechanism of PS subclasses in the impairment of the synapses is based on the inhibition of neuronal development and differentiation and regulation of calcium-dependent signal pathways.

The pathway analysis showed that the revealed signaling pathways of BEB were selected by the KEGG. Amino acid pathways have been found to play a key role in central nervous system, functioning as neurotransmitters, neurochemicals, and energy metabolism regulators. These pathways are believed to be linked to the onset and progression of neurodegenerative disorders [36]. It was discovered that BEB has altered important intermediate metabolites in the pathways associated to aromatic amino acids (phenylalanine, tyrosine, and tryptophan) (Figure 7). The vitamin B6 metabolism pathway observed to be dysregulated in BEB. Studies have reported that dysregulation of vitamin B6 in gut microbiome and serum metabolome are evident among dystonia patients than among controls [12].

## 5. Conclusions

In summary, we generated a nontargeted metabolomic profile in serum between BEB patients and healthy subjects, and we identified 134 differential metabolites for the first time. Then we performed ROC curve analysis and identified several potential biomarkers, including PC (18 : 1(11Z)/24 : 1(15Z)), TG (16 : 0/19 : 0/20 : 0) [iso6], PC (O-22 : 0/22 : 3(10Z,13Z,16Z)), PC (16 : 0/24 : 1(15Z)), PS (16 : 0/22 : 1(11Z)), hexadecyl phosphorodichloridate, methionine sulfoxide, and icotidine. The KEGG pathway enrichment analysis of these differently expressed metabolites in BEB was established. The results suggested that phenylalanine metabolism, phenylalanine, tyrosine and tryptophan biosynthesis, arginine biosynthesis, linoleic acid metabolism, tryptophan metabolism, aminoacyl-tRNA biosynthesis, sphingolipid metabolism, glycosphingolipid biosynthesis, leucine and isoleucine biosynthesis, and vitamin B6 metabolism were responsible for the pathogenesis of BEB. Moreover, antioxidants may become therapeutic targets for BEB due to the role of oxidative stress in the etiology of the disease. The available results are encouraging, considering that the reported biological metabolites will provide novel scientific insights into the pathology and treatment decision of BEB.

## Figures and Tables

**Figure 1:** The workflow of our study.

**Figure 2:** The total ion chromatogram and unsupervised principal component analyses (PCA) scores plot made from the serum samples from BEB patients, healthy controls, and QC groups. The total ion chromatogram of the BEB and healthy controls in the (a) positive and (b) negative ionization modes. (c) PCA scores plot generated from all serum samples in positive ionization mode. (d) PCA scores plot generated from all serum samples in negative ionization mode. BEB: benign essential blepharospasm; QC: quality control.

**Figure 3:** Volcano plot of altered metabolites between the BEB and control groups under positive ionization mode (a), negative ionization mode (b), and combination mode (c). Upregulated metabolites are shown in red, whereas downregulated metabolites are shown in green. BEB: benign essential blepharospasm.

**Figure 4:** Hierarchical clustering heatmap of significantly altered metabolites and the Pair-wise correlation (Spearman) analysis. Hierarchical clustering heatmap of the altered metabolites between the BEB and control groups under positive ionization mode (a), negative ionization mode (b), and combination mode(c). (d) Pair-wise correlation (Spearman) among between serum differential metabolites and clinical parameters. BEB: benign essential blepharospasm.

**Figure 5:** KEGG pathway enrichment analysis of the altered metabolites. KEGG: Kyoto Encyclopedia of Genes and Genomes.

**Figure 6:** ROC curve of the untargeted altered metabolomics according to the criteria (AUC > 0.8). ROC: receiver operating characteristic; AUC: area under the curve.

**Figure 7:** Schematic diagram of the phenylalanine, tyrosine and tryptophan production, phenylalanine metabolism, and tyrosine metabolism pathway. There are still some limitations existed in this study. First of all, we only included 30 BEB patients in our study, and the limited number of BEB patients might not be sufficient to identify the altered metabolic status of BEB patients. So, a larger sample size of BEB patients and cohort are needed to validate our results. Moreover, there is currently a lack of animal and cell models for blepharospasm, so animal and cell-level validation cannot be performed. We have found 134 differential nontargeted metabolites and predicted the possible involvement of signaling pathways of the changed nontargeted metabolites. However, the relationship between these metabolites and BEB is required to be further investigated.

**Table 1:** Basic characteristics of BEB patients and healthy controls.

Parameter	Control	BEB	*p* value
Number (n)	33	30	—
Age (year)	50.06	51.43	0.620
Gender (female/male)	25/8	24/6	0.767
BMI (kg/m^2^)	22.45	22.62	0.872
Course of disease (months)	—	21.03 ± 12.51	—
Jankovic rating scale	—	5 ± 2	—
Blepharospasm disability index	—	2.32 ± 0.97	—

**Table 2:** Diagnostic value of the potential metabolic biomarkers with AUC over 0.8.

Metabolites	AUC	Specificity	Sensitivity	Expression
PC (18 : 1(11Z)/24 : 1(15Z))	1	1	1	-184964
TG (16 : 0/19 : 0/20 : 0) [iso6]	0.99091	0.9	1	63204.1
PC (O-22 : 0/22 : 3(10Z,13Z,16Z))	0.98081	1	0.93939	248438
PC (16 : 0/24 : 1(15Z))	0.97778	0.93333	0.93939	-299051
PS (16 : 0/22 : 1(11Z))	0.91515	0.8	1	-238778
Hexadecyl phosphorodichloridate	0.83535	0.93333	0.72727	51572.7
Methionine sulfoxide	0.82424	0.8	0.78788	-2218584.9
Icotidine	0.80101	0.76667	0.75758	213107

## Data Availability

The data used to support the findings of this study are available from the corresponding authors upon request.

## Supplementary Materials

Supplementary 1 Supplementary Figure 1: PLS-DA and permutation test plots made from the serum samples from BEB patients and healthy controls. (A) PLS-DA scores plot generated from all serum samples in positive ionization mode. (B) PLS-DA scores plot generated from all serum samples in negative ionization mode. (C) Permutation test plot generated from all serum samples in positive ionization mode. (D) Permutation test plot generated from all serum samples in negative ionization mode. PLS-DA: partial least squares-discriminant analysis; BEB: benign essential blepharospasm.

Supplementary 2 Supplementary Figure 2: the ratios of L-kynurenine/tryptophan and tyrosine/phenylalanine in BEB patients and healthy controls. Boxplots are used to display the median and quartiles for the ratios of L-kynurenine to tryptophan (A) and o-tyrosine to phenylalanine (B). *p* values below or below 0.05 are indicated by the symbols ^∗^ and ns.

Supplementary 3 Supplementary Table 1: significantly different metabolites between BEB patients and healthy controls.

Supplementary 4 Supplementary Table 2: significantly altered metabolites at different course of disease.
